The article "Efficacy of Azithromycin plus Glucocorticoid Adjuvant Therapy on Serum Inflammatory Factor Levels and Incidence of Adverse Reactions in Children with Mycoplasma Pneumonia" was retracted in 2023. Reasons: signs of a paper mill; suspected computer-generated content; unreliable results or conclusions; concerns about the data.

# Efficacy of Azithromycin plus Glucocorticoid Adjuvant Therapy on Serum Inflammatory Factor Levels and Incidence of Adverse Reactions in Children with Mycoplasma Pneumonia

**DOI:** 10.1155/2022/1207512

**Published:** 2022-04-04

**Authors:** Yingdong Cao, Binbin Dong, Xuecheng Wang, Chunrong Wang

**Affiliations:** ^1^Department of Pharmacy, Hainan Women and Children's Medical Center, Haikou, Hainan 570100, China; ^2^Department of Pediatrics, Huashan Hospital, Fudan University, Shanghai 200040, China; ^3^Department of Pediatrics, Dongyang Hospital Affiliated to Wenzhou Medical University, Dongyang 322100, China; ^4^Department of Pediatrics, Shanghai Jiading Hospital of Traditional Chinese Medicine, Shanghai 201899, China

## Abstract

**Objective:**

This study was designed to explore the efficacy of azithromycin plus glucocorticoid adjuvant therapy on the levels of serum inflammatory factors and the incidence of adverse reactions in children with mycoplasma pneumonia.

**Method:**

A total of 90 eligible children with mycoplasma pneumonia in our hospital from January 2019 to January 2020 were recruited. They were assigned to receive either azithromycin (control group) or azithromycin plus glucocorticoid (experimental group) according to the order of admission. Outcome measures included clinical efficacy, serum inflammatory factor indicators, lung function, clinical symptom mitigation, length of hospital stay, immune function, incidence of adverse reactions, and psychological status of the eligible children.

**Results:**

Azithromycin plus glucocorticoid was associated with a significantly higher total clinical efficacy compared with azithromycin (*P* < 0.05). No significant differences were found in the serum inflammatory factor indices between the two groups (*P* > 0.05). The children given azithromycin plus glucocorticoid showed lower levels of serum inflammatory factors versus those given azithromycin alone (*P* < 0.001). Azithromycin plus glucocorticoid outperformed the monotherapy of azithromycin in terms of lung function (*P* < 0.001). Children after azithromycin plus glucocorticoid therapy had a faster clinical symptom disappearance and shorter length of hospital stay compared with after azithromycin alone (*P* < 0.001). Azithromycin plus glucocorticoid resulted in higher levels of immune function indices compared with azithromycin alone (*P* < 0.001). Azithromycin plus glucocorticoid was associated with a lower incidence of adverse reactions compared with azithromycin (*P* < 0.05). Lower Children's Depression Inventory (CDI) scores were witnessed in children given azithromycin plus glucocorticoid compared with monotherapy of azithromycin (*P* < 0.001).

The article "Efficacy of Azithromycin plus Glucocorticoid Adjuvant Therapy on Serum Inflammatory Factor Levels and Incidence of Adverse Reactions in Children with Mycoplasma Pneumonia" was retracted in 2023. Reasons: signs of a paper mill; suspected computer-generated content; unreliable results or conclusions; concerns about the data.

**Conclusion:**

Azithromycin plus glucocorticoid in children with mycoplasma pneumonia can effectively improve the clinical indicators of the children with promising efficacy and high safety, which is worthy of promotion and application.

## 1. Introduction

Mycoplasma pneumonia is a common pediatric respiratory disease, which refers to acute inflammation of the lungs and respiratory tract caused by mycoplasma pneumonia infection, with a high prevalence in school-age children and infants [1–3]. The pathogenesis of mycoplasma pneumonia in children is related to autoimmunity and environmental changes, and its clinical manifestations include fever, cough, and upper gastrointestinal infection. Ineffective or delayed treatment may result in Guillain–Barré syndrome, nephritis, and complications, which severely compromises the health of children and hinders the growth and development of children [4–6]. At present, clinical treatment is mainly drug therapy to suppress disease progression, control infection, and improve ventilation in children. As a macrolide antibiotic with wide clinical application, azithromycin can relieve the clinical symptoms of children, though the therapeutic effect of its single medication fails to meet the clinical expectations with a poor safety profile [7, 8]. It has been clinically found that azithromycin plus glucocorticoid yields a significant clinical effect on the treatment of mycoplasma pneumonia in children. Accordingly, to further explore the effect of azithromycin plus glucocorticoids on the serum inflammatory factor levels and the incidence of adverse reactions in children with mycoplasma pneumonia, 90 cases of mycoplasma pneumonia in our hospital from January 2019 to January 2020 were recruited. The results are as follows.

## 2. Materials and Methods

### 2.1. General Materials

A total of 90 children with mycoplasma pneumonia in our hospital from January 2019 to January 2020 were recruited and were assigned to either a control group or an experimental group according to the order of admission.

### 2.2. Inclusion Criteria

The inclusion criteria were as follows: ① age range: 1.5–4.5 years; ② after admission, routine laboratory examinations, chest X-rays, lung CTs, and other related special examinations were performed, and their diagnoses were all in line with the diagnostic criteria for mycoplasma pneumonia by *Respiratory Group of the Pediatric Branch of the Chinese Medical Association*; ③ this study was approved by the hospital ethics committee (approval no. 2018–22901), and the children and their families were informed of the purpose and process of the study and provided written informed consent.

### 2.3. Exclusion Criteria

The exclusion criteria were as follows: ① children with severe liver and kidney disease; ② children with drug allergies; ③ children with serious cardiovascular and cerebrovascular diseases; ④ children with autoimmune diseases.

The article "Efficacy of Azithromycin plus Glucocorticoid Adjuvant Therapy on Serum Inflammatory Factor Levels and Incidence of Adverse Reactions in Children with Mycoplasma Pneumonia" was retracted in 2023. Reasons: signs of a paper mill; suspected computer-generated content; unreliable results or conclusions; concerns about the data.

### 2.4. Methods

The control group was treated with intravenous infusion of azithromycin injection (manufacturer: Yabao Pharmaceutical Group Co., Ltd.; NMPA approval number: H20051466; specification: 2 ml: 0.1 g). The azithromycin injection 10 mg kg^−1^ d^−1^ was added into 250 ml of 0.9% sodium chloride injection, with the concentration of 1.0 mg/ml–2.00 mg/ml and the infusion time of >60 min, and the maximum dose was less than 500 mg per day. The dose was determined based on the children body weight, and the treatment spanned 14 d.

The experimental group was given azithromycin plus glucocorticoid adjuvant intravenous instillation therapy. Methylprednisolone injection (manufacturer: Pfizer Manufacturing Belgium NV, NMPA approval number: 20170199, specification: 0.5 g^*∗*^1 bottle/box) 0.3 mg kg^−1^ d^−1^ was diluted by 2 mg–20 mg + 5% glucose injection for treatment. Repeated administration was given every 3 h–5 h, and the interval of continuous administration should be maintained within 72 h. The dose was determined based on the children body weight, and the treatment spanned 14 d.

The above treatment was carried out in our hospital. The detailed process is shown in Figure 1.

### 2.5. Outcome Measures

Clinical efficacy: marked effective: the symptoms disappear, and the body temperature and the physical signs return to normal; effective: the symptoms are significantly relieved with a decrease of the body temperature, but the physical signs are not fully recovered; ineffective: the above symptoms remain static or aggravated.

The fasting venous blood of the two groups of children was collected in the early morning and centrifugated to obtain the supernatant. All serum samples were placed at −80°C, and the serum inflammatory factors including C-reactive protein (CRP), interleukin-8 (IL-8), and matrix metalloproteinase-9 (MMP-9) were determined strictly according to the ELISA kit instructions and operating procedures.

The lung function indexes including respiratory rate (RR), peak volume ratio (VPTFF/tE), and peak time ratio (TPTFF/tE) were recorded.

The time to clinical symptoms disappearance and the length of hospital stay between the two groups of children were compared.

The immune function indexes of the two groups of children after treatment were compared. Fasting venous blood was collected from all children, and 2 mL of blood samples were anticoagulated with ethylenediaminetetraacetic acid. The flow cytometer (manufacturer: German Partec; model: CyFlow® Ploidy Analyser) was used to determine the levels of CD4, CD8, and CD4/CD8 in the T lymphocyte subsets of the two groups of children.

The article "Efficacy of Azithromycin plus Glucocorticoid Adjuvant Therapy on Serum Inflammatory Factor Levels and Incidence of Adverse Reactions in Children with Mycoplasma Pneumonia" was retracted in 2023. Reasons: signs of a paper mill; suspected computer-generated content; unreliable results or conclusions; concerns about the data.

The incidence of adverse reactions between the two groups was compared. Adverse reactions included stomach aches, nausea, and vomiting.

The “Children's Depression Inventory (CDI)” [9] was used to evaluate the psychological status of the eligible children. The scale has a total of 54 points. The higher the score, the more severe the depression of the child.

### 2.6. Statistical Processing

The data processing software selected in this research was SPSS20.0, and GraphPad Prism 7 (GraphPad Software, San Diego, USA) was used to plot the graphs. The counting data adopted the *χ*^2^ test and were expressed by (*n* (%)), and the measurement data were expressed by $\left(\bar{x}\pm s\right)$ and analyzed by the *t*-test. *P* < 0.05 indicates that the difference is statistically significant.

## 3. Results

### 3.1. Baseline Data

There were no significant differences in gender, average age, average course of the disease, BMI, average body temperature, and place of residence between the two groups of children (*P* > 0.05) (Table 1).

### 3.2. Clinical Efficacy

Azithromycin plus glucocorticoid was associated with a significantly higher total clinical efficacy compared with azithromycin (*P* < 0.05) (Table 2).

### 3.3. Serum Inflammatory Factors

No significant differences were found in the serum inflammatory factor indices between the two groups (*P* > 0.05). The children given azithromycin plus glucocorticoid showed lower levels of serum inflammatory factors compared with those given azithromycin alone (*P* < 0.001) (Table 3).

### 3.4. Lung Function

Azithromycin plus glucocorticoid outperformed the monotherapy of azithromycin in terms of lung function (*P* < 0.001) (Table 4).

### 3.5. Disappearance Time of Clinical Symptoms and Length of Hospital Stay

Children after azithromycin plus glucocorticoid therapy had a faster clinical symptom disappearance and shorter length of hospital stay compared with after azithromycin alone (*P* < 0.001) (Table 5).

### 3.6. Immune Function

Azithromycin plus glucocorticoid resulted in higher levels of immune function indices compared with azithromycin alone (*P* < 0.001) (Table 6).

### 3.7. Incidence of Adverse Reactions

Azithromycin plus glucocorticoid was associated with a lower incidence of adverse reactions compared with azithromycin (*P* < 0.05) (Figure 2).

### 3.8. CDI Scores

Lower Children's Depression Inventory (CDI) scores were witnessed in children given azithromycin plus glucocorticoid compared with monotherapy of azithromycin (*P* < 0.001) (Figure 3).

The article "Efficacy of Azithromycin plus Glucocorticoid Adjuvant Therapy on Serum Inflammatory Factor Levels and Incidence of Adverse Reactions in Children with Mycoplasma Pneumonia" was retracted in 2023. Reasons: signs of a paper mill; suspected computer-generated content; unreliable results or conclusions; concerns about the data.

## 4. Discussion

In recent years, with environmental pollution and changes in lifestyle, the incidence of mycoplasma pneumonia in children has been witnessing a trend of increase [10, 11]. Relevant literature shows that mycoplasma pneumonia in children mostly occurs in autumn and winter, and the prevalence in children over 5 years old is 20.94%, with the characteristics of a heavy, prolonged, and recurrent disease. Given the underdeveloped immune function in children, delayed or ineffective treatment can be life-threatening [12–14]. Currently, clinical treatment is mainly based on drug therapy. Azithromycin, as a widely used antibiotic drug in clinical practice, is featured by a good absorption and long half-life, which effectively improves the clinical indices and the immunity of children. However, the efficacy of single-drug treatment fails to meet the expectations [15, 16]. Glucocorticoids are considered effective in inhibiting the development of children's disease and boosting the rapid recovery of the disease.

In the present study, azithromycin plus glucocorticoid was associated with a significantly higher total clinical efficacy compared with azithromycin (*P* < 0.05), indicating that compared with a single medication, combined medication treatment possesses a more significant efficacy. Previous studies pointed out that inflammatory factors play an important role in the formation of mycoplasma pneumonia in children [17–19]. The invasion of bacteria in the child's lungs may generate corresponding toxins to stimulate the lung macrophages to release inflammatory factors, thereby triggering an inflammatory response. As common indicators of inflammatory factors, the levels of serum CRP, IL-8, and MMP-9 can directly reflect the inflammatory state of children [20, 21]. As an acute phase response protein, CRP will increase rapidly after tissue injury. Therefore, clinical testing of CRP is contributory to the early disease detection of the child. As a chemotactic cytokine, IL-8 has been recognized for its role in the pathological process of children. The level of the MMP-9 index represents the specific changes in the child's condition [22]. Herein, the children given azithromycin plus glucocorticoid showed lower levels of serum inflammatory factors compared with those given azithromycin alone (*P* < 0.05), indicating that azithromycin plus glucocorticoid can effectively mitigate the inflammatory responses in children. In addition, azithromycin plus glucocorticoid outperformed the monotherapy of azithromycin in terms of lung function, clinical symptom disappearance, and length of hospital stay (*P* < 0.05), which suggests that the combined medication regimen features a quick effect and can effectively alleviate the symptoms of pneumonia, improve the lung function of the children, and is conducive to the rapid recovery of the children.

The article "Efficacy of Azithromycin plus Glucocorticoid Adjuvant Therapy on Serum Inflammatory Factor Levels and Incidence of Adverse Reactions in Children with Mycoplasma Pneumonia" was retracted in 2023. Reasons: signs of a paper mill; suspected computer-generated content; unreliable results or conclusions; concerns about the data.

With a high level of intracellular concentration and bioavailability, azithromycin is the mainstay for the clinical treatment of mycoplasma pneumonia in children. As a glucocorticoid, methylprednisolone injection possesses antitoxic, anti-inflammatory, and antishock effects, which can mitigate vasodilation, stabilize the lysosome membrane, inhibit phagocytosis, and substantially treat inflammation caused by the abnormal immune system [23, 24]. In the present study, azithromycin plus glucocorticoid resulted in higher levels of immune function indices compared with azithromycin alone (*P* < 0.05), indicating that azithromycin plus glucocorticoid adjuvant therapy can prominently enhance the immunity of children. In most cases, children may experience anxiety and fear during treatment. Ineffective treatment measures for children may increase their pressure, which compromises the prognosis. Herein, the CDI score of the experimental group after treatment was significantly lower than that of the control group (*P* < 0.05), indicating that the combination treatment can effectively alleviate the children's negative emotions and promote the recovery of the disease. The results of this experiment also showed a lower incidence of adverse reactions of azithromycin plus glucocorticoid compared with azithromycin (*P* < 0.05), which was consistent with the results of Rovani et al. [25], whose article pointed out that “the total incidence rate of adverse reactions in the observation group is 8.0% (4/50), which is lower than 14.0% (7/50) of the control group (*x*^2^ = 4.245, *P*=0.034).” It indicates a higher safety of azithromycin plus glucocorticoid therapy compared with monotherapy of azithromycin.

## 5. Conclusion

In summary, the application of azithromycin plus glucocorticoid adjuvant therapy in children with mycoplasma pneumonia can effectively improve clinical efficacy, can mitigate inflammatory responses, and features a high safety profile, so it is worthy of promotion and application.

## Figures and Tables

**Figure 1:** Technical streamline diagram.

**Figure 2:** Comparison of the incidence rate of adverse reactions between the two groups (*n* (%)). *Note.* Black represents stomachache; red represents nausea; yellow represents vomiting; white represents no adverse reactions. The composition of adverse reactions in the experimental group was 1 case of stomachache (2.22%), 1 case of nausea (2.22%), 1 case (2.22%) of vomiting, and 42 cases (93.33%) of no adverse reactions occurred, and totally 3 cases of adverse reactions (6.67%). The composition of adverse reactions in the control group was 3 cases of abdominal pain (6.67%), 4 cases of nausea (8.89%), 4 cases (8.89%) of vomiting, and 34 cases (75.56%) of no adverse reactions occurred, and the total number of adverse reactions was 11 cases (24.44%). There was a significant difference in the incidence rate of adverse reactions between the two groups (*x*^2^ = 5.414, *P* < 0.05).

The article "Efficacy of Azithromycin plus Glucocorticoid Adjuvant Therapy on Serum Inflammatory Factor Levels and Incidence of Adverse Reactions in Children with Mycoplasma Pneumonia" was retracted in 2023. Reasons: signs of a paper mill; suspected computer-generated content; unreliable results or conclusions; concerns about the data.

**Figure 3:** Comparison of CDI scores between the two groups $\left(\bar{x}\pm s\right)$. *Note.* The abscissa represents before and after treatment, respectively, and the ordinate represents CDI score; the CDI scores of the experimental group before and after treatment were (27.25 ± 4.13) points and (6.32 ± 1.25) points, respectively; the CDI scores of the control group before and after treatment were (27.24 ± 4.15) points and (13.56 ± 2.76) points, respectively; ^*∗*^ indicates that there was a significant difference in the CDI scores of the experimental group before and after treatment (*t* = 32.538, *P* < 0.001); ^*∗∗*^ indicates that there was a significant difference in the CDI scores of the control group before and after treatment (*t* = 18.413, *P* < 0.001); ^*∗∗∗*^ indicates that there was a significant difference in CDI scores between the two groups of patients after treatment (*t* = 16.029, *P* < 0.001).

**Table 1:** Comparison of general information between the two groups of children (*n* (%)).

	Experimental group (*n* = 45)	Control group (*n* = 45)	*χ* ^2^ or *t*	*P*
Gender			0.178	0.673
Male	23 (51.11)	21 (46.67)		
Female	22 (48.89)	24 (53.33)		

Average age (year-old)	3.07 ± 0.31	3.11 ± 0.27	0.147	0.883
Average course of disease (d)	8.12 ± 2.13	8.11 ± 2.11	0.022	0.982
BMI (kg/m^2^)	17.55 ± 3.42	17.49 ± 3.31	0.085	0.933
Average body temperature (°C)	39.51 ± 0.78	39.53 ± 0.79	0.121	0.904
Place of residence			0.182	0.670
Urban	25 (56.25)	27 (50.00)		
Rural	20 (43.75)	18 (50.00)		

**Table 2:** Comparison of clinical efficacy between the two groups (*n* (%)).

Group	*n*	Markedly effective	Effective	Not effective	Total effective rate
Experimental group	45	55.56% (25/45)	37.78% (17/45)	6.67% (3/45)	93.33% (42/45)
Control group	45	42.22% (19/45)	28.89% (13/45)	28.89% (13/45)	71.11% (32/45)
*χ* ^2^					7.601
*P*					<0.05

**Table 3:** Comparison of serum inflammatory factors between the two groups $\left(\bar{x}\pm s\right)$.

Group	*n*	CRP (mg/L)		IL-8 (pg/L)		MMP-9 (U/L)	
		Pretreatment	Posttreatment	Pretreatment	Posttreatment	Pretreatment	Posttreatment
Experimental	45	25.88 ± 2.36	2.11 ± 0.57	521.35 ± 61.36	171.15 ± 28.27	272.25 ± 53.53	149.27 ± 21.35
Control	45	25.85 ± 2.35	5.39 ± 0.25	520.37 ± 61.39	225.36 ± 35.35	273.28 ± 53.49	187.41 ± 32.68
*t*		0.060	35.351	0.076	8.034	0.091	6.554
*P*		0.952	<0.001	0.939	<0.001	0.928	<0.001

The article "Efficacy of Azithromycin plus Glucocorticoid Adjuvant Therapy on Serum Inflammatory Factor Levels and Incidence of Adverse Reactions in Children with Mycoplasma Pneumonia" was retracted in 2023. Reasons: signs of a paper mill; suspected computer-generated content; unreliable results or conclusions; concerns about the data.

**Table 4:** Comparison of lung function indexes between the two groups $\left(\bar{x}\pm s\right)$.

Group	*n*	RR (number of times/min)		V_PTFF_/*t*_E_ (%)		T_PTFF_/*t*_E_ (%)	
		Pretreatment	Posttreatment	Pretreatment	Posttreatment	Pretreatment	Posttreatment
Experimental	45	70.33 ± 7.15	25.11 ± 6.53	13.35 ± 0.95	31.23 ± 3.27	11.37 ± 1.28	28.53 ± 3.19
Control	45	70.36 ± 7.17	24.27 ± 6.35	13.37 ± 0.94	18.26 ± 3.13	11.38 ± 1.31	15.41 ± 2.98
*t*		0.044	21.059	0.100	19.221	0.037	20.161
*P*		0.952	<0.001	0.920	<0.001	0.971	<0.001

**Table 5:** Comparison of the disappearance time of clinical symptoms and hospital length of stay between the two groups $\left(\bar{x}\pm s\right)$.

Group	*n*	Disappearance time of cough	Fever clearance time	Disappearance time of pulmonary rales	Length of stay
Experimental group	45	3.02 ± 0.45	1.68 ± 0.35	4.37 ± 1.25	5.36 ± 1.63
Control group	45	5.61 ± 1.17	3.72 ± 0.61	6.99 ± 1.54	8.01 ± 1.41
*t*		13.859	19.459	8.861	8.248
*P*		<0.001	<0.001	<0.001	<0.001

**Table 6:** Comparison of immune function indexes between the two groups$\left(\bar{x}\pm s\right)$.

Group	*n*	CD4 (%)	CD8 (%)	CD4/CD8
Experimental group	45	38.27 ± 8.02	21.03 ± 6.31	1.73 ± 0.52
Control group	45	30.25 ± 7.93	28.03 ± 7.27	1.27 ± 0.43
*t*		4.770	4.878	4.573
*P*		<0.001	<0.001	<0.001

## Data Availability

All data generated or analyzed during this study are included in this published article.
